# Pathological, Histological, and Molecular Based Investigations Confirm Novel *Mycobacterium bovis* Infection in *Boselaphus tragocamelus*

**DOI:** 10.1155/2022/7601463

**Published:** 2022-06-02

**Authors:** Riaz Hussain, Adil Jamal, Zulfiqar Ahmed, Bahaeldeen Babiker Mohamed, Abu Baker Siddique, Iahtasham Khan, Muhammad Khalid Mansoor, Xiaoxia Du, Ahrar Khan

**Affiliations:** ^1^Department of Pathology, Faculty of Veterinary and Animal Sciences, The Islamia University of Bahawalpur, 63100, Pakistan; ^2^Sciences and Research, College of Nursing, Umm Al Qura University, 715 Makkah, Saudi Arabia; ^3^Department of Food Science and Technology, Faculty of Agriculture and Environment, The Islamia University of Bahawalpur, 63100, Pakistan; ^4^Institute of Environment Natural Resources, The National Centre of Research, Khartoum, Sudan; ^5^Department of Microbiology, Government College University, Faisalabad 38000, Pakistan; ^6^Section of Epidemiology and Public Health, University of Veterinary and Animal Sciences, Lahore, Sub-Campus Jhang, Pakistan; ^7^Department of Microbiology, Faculty of Veterinary and Animal Sciences, The Islamia University of Bahawalpur-63100, Pakistan; ^8^Shandong Vocational Animal Science and Veterinary College, Weifang 261061, China; ^9^Faculty of Veterinary Science, University of Agriculture, Faisalabad 38040, Pakistan

## Abstract

*Mycobacterium bovis* (*M. bovis*) being the main cause of animal tuberculosis is a complex infectious agent and can be a cause of zoonotic tuberculosis zoonosis in public health. To date, the uncommon infection in public health due to *M. bovis* still is a great challenge to both veterinary and medical professions and requires a careful diagnosis and confirmation of the bacterium. Therefore, this study for the first time reports the clinical, gross, histopathological, and molecular based confirmation of *M. bovis* infection in wildlife animals (nilgai). Prior to death, the morbid animal showed severe pneumonic ailments like moist cough, thick nasal exudates, and dyspnoea. At necropsy, enlargement of mandibular cervical and mesenteric lymph nodes was observed. Different macroscopic lesions such as congestion and hyperaemia, creamy white and catarrhal exudates in trachea, consolidation, grey and red hepatisation of lungs, and micro- and macrogranulomatous tubercles containing caseous materials in lungs were observed. The heart of morbid animal showed congestions, myocarditis, and a copious amount of straw-colored fluid in the pericardial sac. At the microscopic level, lungs indicated granulomatous inflammatory response, presence of multinucleated giant cells, fibrosis, and punctuation of alveoli with chronic inflammatory cells. Histopathological examination of various sections of the heart of the infected animal showed chronic inflammatory response consisting of chronic inflammatory cells like monocyte, lymphocytes, and fibroblasts along with noncalcified eosinophilic materials. At the molecular level, *M. bovis* infection was confirmed in various tissues like the heart, lungs, cervical, and mesenteric lymph nodes in morbid animals. In conclusion, based on our results, it can be suggested that more molecular based epidemiological studies are crucial to know the exact cause of pulmonary and cervical tuberculosis in wild animals.

## 1. Introduction

The majority of newly emerging human diseases are caused by zoonotic diseases. Furthermore, 71% of newly emerging diseases are either derived from wildlife or have an epidemiologically significant animal host [1]. Many of the diseases that infect domestic animals can also infect wild animals, and transmission between domestic animals and wildlife can occur in both directions. The primary occurrence, however, was frequently the spread of disease from domestic animals to wildlife. *Mycobacterium bovis*, the causal agent of tuberculosis in cattle and most other mammals, wild or domestic, is one such pathogen [2]. Importantly, it has a wide spectrum of hosts including humans [3].

*Mycobacterium tuberculosis* of the family Mycobacteriaceae is Gram-positive and rod-shaped and causes tuberculosis in mammals.*Mycobacterium bovis* (bovine tuberculosis), *M. caprae* (caprine tuberculosis), *M. pinnipedii*, *M. orygis*, and *M. microti* are reported in animals [4]. *Mycobacterium caprae*, *M. pinnipedii*, and *M. orygis* are classified as subspecies of *M. bovis*. Two other organisms, *M. tuberculosis* and *M. africanum*, are found in humans but infect animals infrequently [4]. A few countries (for example, Australia, Iceland, Greenland, Singapore, several European countries, and Israel) are completely free of *M. bovis*, although infected cattle herds are now rare in Europe, Canada, United States, New Zealand, and other countries.

The majority of data on zoonotic mycobacteria transmission is evidenced by investigations on *M. bovis* [4]. Depending on the areas, where it has localized, the causal organism may be identified in respiratory secretions, exudates/secretions from lesions (e.g., draining lymph nodes, certain skin lesions), urine, feces, milk, vaginal discharge, and semen. *Mycobacterium bovis* is more likely to be transferred when the respiratory system gets infected and during the late stages of the disease with widespread lesions [4]. The extent to which an infected host brings itself or its excretions into close contact with other vulnerable hosts, including members of the same species, is determined by host ecology and behaviour [5].

Prevalence alludes not only to the quantity of diseased animals in a given community but also to their geographic and temporal distribution [5]. Multiple species are epidemiologically linked in several countries with suspected or confirmed *M. bovis* wildlife animals, which may involve multiple hosts and different transmission routes [6]. In Pakistan, different species of livestock animals including large ruminants (camel, cattle, and buffaloes) and small ruminants (sheep and goat) are particularly kept for milk and meat purposes [7–10]. These animals are usually and mainly reared under tropical and subtropical conditions in the country. Epidemiological studies in Pakistan have reported the prevalence of contagious and zoonotic bacteria [11–17], parasites [18], and viral diseases [19]. Among various zoonotic diseases, tuberculosis due to *M. bovis* is a fatal problem for dairy and wild animals [20–22]. *Mycobacterium bovis* infection causes huge economic losses in terms of reduced milk yield, increased cost of treatment and control strategies, culling of infected animals, and limiting the international trade of dairy animals and their products [23].

Studies have indicated that in several developing countries, *M. bovis* acts as an endemic threat [24, 25] and has been reported in free-ranging carnivores and wild animals [26, 27]. Earlier studies have reported a 5.75% prevalence of *M. bovis* infection in cattle and buffalo while 4% in humans [28, 29]. Recently, in Pakistan, 5.88% of *M. bovis* infection has been recorded in different districts of Pakhtunkhwa [23]. Higher prevalence of *M. bovis* infection in buffaloes (8.48%) reared at various livestock farms [30] and in cattle (11.71%) of different private farms has been recorded [31]. Several studies in Pakistan have determined an increased prevalence *M. bovis* infection such as 12.72% [32], 11.3% [33], 10.6% [34], 7.47% [35], and 9.6% in dairy animals [36]. A lower prevalence (2.2-3%) of *M. bovis* infection in buffaloes kept at different locations in Punjab has also been documented [30, 37]. Previously, scanty information could be found regarding the prevalence of bovine tuberculosis in different zoo animals including Bovidae and Cervidae [38].

The exact mechanisms of spread and transmission of *M. bovis* to wildlife animals still remain unclear. However, the wild animals may get these infections directly via close contact with scavengers or indirectly through contamination of the environment or ingestion of infected products. Few reports are available about bovine tuberculosis in wild animals kept at various zoological parks and different zoos in Pakistan [19].

Tuberculosis is commonly diagnosed by isolating the organism from the sputum, milk, feces, and other bodily fluids [39]. Tuberculosis is commonly detected using direct smear microscopy with the fluorescent acid-fast staining technique and Ziehl-(ZN) Neelsen's staining of clinical samples [39]. Although culturing on selective media provides a confirmed *Mycobacterium* diagnosis, the main disadvantage of this approach is the slow bacterial growth [40]. Using polymerase chain reaction (PCR) amplification of the *Mycobacterium* DNA, it is possible to make a rapid diagnosis of *Mycobacterium* from clinical samples. PCR is a more precise and reliable method for rapid diagnosis, with substantially higher sensitivity and specificity than bacterial culture [40]. It is necessary to comprehend the involvement of wildlife in the epidemiology of *M. bovis* infection.

This study is aimed at studying necropsy lesions and histopathological findings of tuberculosis due to *M. bovis* in nilgai. *Mycobacterium bovis* detection was further confirmed using PCR. Regular livestock and wildlife screening will help prevent *M. bovis* transmission to other animals.

## 2. Materials and Methods

### 2.1. Ethical statement

The technical and ethical committee constituted by the Department of Pathology, Faculty of Veterinary and Animal Sciences, the Islamia University of Bahawalpur, Pakistan, approved the protocol of the postmortem study of nilgai.

### 2.2. Study Location and Animals

The current study included two animals that suddenly died at Bahawalpur Zoo, Punjab, Pakistan. Both the animals were kept together under tropical and subtropical environmental conditions. History from the concerned veterinarian and curator of the zoo revealed that a male nilgai become sick and exhibited different clinical signs like anorexia, being reluctant to move, depression, dyspnea, lethargy, disorientation, and coughing while the female died without any signs of respiratory infections and exhibited increased watery fluid from mouth and disorientation. These animals were offered seasonal green fodder and grain (0.5 kg) daily. In one case, the persistent cough was a prominent clinical sign observed early in the morning and during the late evening. In spite of extensive care, management practices, and treatment therapy, the animals died. The necropsy was performed after half an hour of death to determine the possible cause of death.

### 2.3. Necropsy and Histopathological Investigation

Prior to complete skinning and abdominal opening, the nilgai were carefully observed for external lesions. The nilgai were quite normal and had fair body conditions. At necropsy, the external examination showed severe congested nasal passages and thick nasal discharge before skinning in the male while enlarged and swollen cervical and mandibular lymph nodes in the female. After thorough and complete external observation, the dead animals were dissected and opened to know any internal lesions.

### 2.4. Sample Collection and Histopathology Studies

The visceral organs showing abnormal lesions such as the lungs and heart were removed and immediately fixed in 10% neutral buffered formalin solutions for histological changes [10]. For histopathological observations, various tissues from the lungs and heart were embedded in paraffin wax, and about 5 *μ*m-thick sections were stained with haematoxylin and eosin (H&E) stains [41].

### 2.5. Genetic Analysis

For bacilli confirmation, different tissue samples having lesions, e.g., the lungs, heart, mesenteric, and cervical lymph nodes, were used for bacterial DNA extraction and confirmation of suspected cause [42]. Genomic DNA was extracted from samples using the GeneJET Genomic DNA Extraction kit (Cat# K0721, Thermo Scientific™, USA) following the manufacturer's guidelines. The gene-specific primer targeting the JB21 and JB22 genes (sense JB21; 5′-TCGTCCGCTGATGCAAGTGC-3′, antisense JB22; 5′-CGTCCGCTGACCTCAAGAAG-3′) was used for the genomic amplification of *M. bovis* in samples [43]. The PCR was performed in a thermocycler (Bio-Rad, T100 Thermal Cycler, USA) using the master mixture (Cat # 0171, Invitrogen, USA). The PCR product was run on 1% agarose gel for electrophoreses and visualized through the Gel Documentation System (GelDoc Go System, Bio-Rad, USA).

## 3. Results and Discussion

### 3.1. Disease Onset (Signs and Symptoms)

In wildlife, particularly ungulates and free-ranging species, the diagnosis of *M. bovis* infection mainly involves culturing of an infectious microbial agent, postmortem lesions, and tissue studies [21]. It has been determined that wild animals can get the infection by preys or scavenged carcasses and disseminate the infection to other animals. Therefore, continuous monitoring and diagnosis of *M. bovis* are crucial to controlling its spread in wildlife, domestic animals, and public health. The morbid nilgai exhibited different nonspecific clinical signs like cough, dyspnoea, and thick nasal exudates prior to death. Previously, no clinical signs of tuberculosis including cough have been observed in experimentally induced captive wild animals [44]. Tuberculosis in wild animals is frequently diagnosed at necropsy after natural death, with no prior suspicion of tuberculosis. Gross lesions may be substantial, covering whole organs in one or both cavities; nevertheless, the anatomical sites of the lesions, the level of pathological involvement, and the nature of nodular structures with some conjunctiva necrosis are frequently present before unthriftiness is often obvious [45].

### 3.2. Disease Progression and Development

During necropsy, our study reported severely congested trachea with creamy white catarrhal exudate. The lungs exhibited small granulomatous tubercles, severe consolidation, and grey and red hepatisation, and cut sections showed a creamy white caseous material (Figure 1). At necropsy, enlarged mandibular, cervical, and mesenteric lymph nodes are packed with caseated and calcified exudate (Figure 2). So far, no published report is available about these lesions in nilgai due to *M. bovis* infection. Lesions in cervids, thoracic cavities, and lymph nodes may be purulent, while others may be dry, depending on where they are located in the animal's body [46, 47]. However, few studies have observed similar pneumonic lesions due to *M. bovis* infection in wild animals [48]. Oryx, nilgai, and stable antelope tumors are strikingly similar to those found in other Bovidae species. There is no evidence of connective tissue involvement in the nodular areas of caseation and epithelioid cells [49]. However, *M. bovis* infection has also been detected in lymph nodes of buffaloes [50], mesenteric lymph nodes [51], and cervical lymphadenitis [52].

### 3.3. Histopathology

At a microscopic level, the lungs indicated congestion, emphysema, infiltration of chronic inflammatory cells, granulomatous inflammation, multinucleated giant cells, fibrosis, and alveoli punctuated with chronic inflammatory cells (Figure 3). Our observations regarding different microscopic lesions in lungs of nilgai, similar lesions due to bovine tuberculosis, including lymphohistiocytic inflammatory and necrotic debris in bears [21], granulomatous lesions comprising caseation surrounded by plasma cells epithelioid, lymphocytes, multinucleated giant cells, and fibrous capsule in rhinoceros and dairy cattle have been investigated earlier [11, 44, 53, 54]. Furthermore, similar histopathological lesions due to experimental infection induced by *M. bovis* in the lungs of deer and cattle have been observed previously [55]. In our findings, the heart of nilgai was extensively enlarged, hyperaemic, and dark in color with a huge amount of straw-colored fluid in the pericardial sac (Figure 4). The Histopathological observation of heart sections showed a caseous material in lamellar arrangement, immature and mature tubercles, infiltration of mononuclear cells, micronodules, and calcified exudates surrounded by fronts of monocytes, fibroblast, macrophage, and fibrocyte (Figure 4). Moreover, heart tissues showed the presence of few neutrophils, eosinophilic noncellular oedematous and homogeneous fluid. No report is available about the different lesions in heart of infected animals due to tuberculosis. Previously, chronic microscopic lesions in the kidneys, liver, and lungs of nilgai that died from bovine tuberculosis have also been observed [56]. The heart lesions observed in Nilgai due to *M. bovis* might be the due release of nucleases and proteases in multiple chronic inflammatory cells comprising macrophages, epithelioid cells, plasma cells, and neutrophils resulting to liquefaction [57]. However, similar pathological lesions in the liver of infected animals have been observed [11]. Therefore, the prevalence of *M. bovis* infection in wild animals and the increasing frequency of the infectious agent draw huge attention for its regular screening not only in domestic animals but also in wildlife in captivity.

### 3.4. Molecular Confirmation

Genotype approaches have been beneficial in epidemiological investigations to determine the source of infection [58–60]. PCR assays are the most promising alternative method for tuberculosis detection with regard to specificity and sensitivity [61, 62]. In a range of biological samples, such as tissue, blood, and nasal exudates, PCR techniques have been successfully used to diagnose *M. bovis* [63, 64]. Our study reported the JB21 and JB22 amplified regions of the *Mycobacterium* genome (Figure 5). Similar genetic analyses have been shown to be very effective in detecting *M. bovis* DNA isolates from blood samples, with 100% accuracy when compared to the traditional microbiological method [65, 66]. In line with the global effort to halt the tuberculosis disease outbreak, it is critical to determine the true burden of zoonotic tuberculosis, particularly in the low- and middle-income countries, where cattle-control programs may be marginal or nonexistent. The epidemiology of tuberculosis can be better understood by combining traditional disease-tracing investigation with molecular typing, which can reveal the role played by various hosts in the spread of disease infection.

## 4. Conclusion and Future Perspective

In recent years, the frequency of tuberculosis in zoo animals has grown, which may be related to the closer confinement of several wild species in one location. The ease and regularity with which organisms transmit from animal to human attract increasing attention to zoonotic relevance. In this regard, there is an urgent need for ongoing research into this disease in both captive and free-roaming wild animals. Only one isolate from nilgai was analyzed in this study, but a more detailed study with a larger sample size would be preferable to improve the transmission routes and the pathology of *M. bovis*. It is also critical to investigate the incidence of *M. bovis* in other animals in developing countries like Pakistan.

## Figures and Tables

**Figure 1:** Photograph lungs of Nilgai showing (a) multifocal tubercles and red hepatisation, (b, c) cut sections exhibiting creamy white exudates, and (d) severe emphysema in the lungs of nilgai that died from *M. bovis* infection.

**Figure 2:** Necropsy of Nilgai showing (a, b) caseated exudate and calcified lymph nodes in opened neck region (arrows) and (c, d) enlarged, caseated exudate, and calcified mesenteric lymph nodes (arrows).

**Figure 3:** Photomicrograph of the lungs of nilgai of tuberculosis showing (a) severe edema, congestion, small foci of abscess, (b) fibrosis, ruptured interalveolar septa, hyperplasia of pneumocyte, (c) micronodules, chronic inflammatory cells in alveolar spaces and obliteration of alveoli, and (d) extensive exudate containing fibroblast, macrophage, monocytes, and thick interlobular septa (H&E; 200X).

**Figure 4:** Photograph of the heart of Nilgai showing (a) congestion and presence of straw-colored fluid in the cardiac cavity and (b) severe inflammatory exudates, fibrosis, and calcified material surrounded by chronic inflammatory cells and immature tubercles in the heart of nilgai that died from *M. bovis* infection. (H&E; 400X).

**Figure 5:** Confirmation of *Mycobacterium bovis* by PCR (500 bp). Lane L shows DNA ladder (100 bp), lanes 1-4 show PCR positive samples, and lane B with no band shows negative control.

## Data Availability

All the data relevant to this study is mentioned in the manuscript. There is no supplementary data.
